The article "Inertial-Based Human Motion Capture: A Technical Summary of Current Processing Methodologies for Spatiotemporal and Kinematic Measures" was published in 2021. Journal: Appl Bionics Biomech.

# Inertial-Based Human Motion Capture: A Technical Summary of Current Processing Methodologies for Spatiotemporal and Kinematic Measures

**DOI:** 10.1155/2021/6628320

**Published:** 2021-03-26

**Authors:** Benjamin R. Hindle, Justin W. L. Keogh, Anna V. Lorimer

**Affiliations:** ^1^Faculty of Health Sciences and Medicine, Bond University, Gold Coast 4226, Australia; ^2^Sports Performance Research Institute New Zealand (SPRINZ), AUT Millennium Institute, AUT University, Auckland 0632, New Zealand; ^3^Cluster for Health Improvement, Faculty of Science, Health, Education and Engineering, University of Sunshine Coast, Sunshine Coast 4556, Australia; ^4^Kasturba Medical College, Mangalore, Manipal Academy of Higher Education, Manipal, Karnataka 576104, India

## Abstract

Inertial-based motion capture (IMC) has been suggested to overcome many of the limitations of traditional motion capture systems. The validity of IMC is, however, suggested to be dependent on the methodologies used to process the raw data collected by the inertial device. The aim of this technical summary is to provide researchers and developers with a starting point from which to further develop the current IMC data processing methodologies used to estimate human spatiotemporal and kinematic measures. The main workflow pertaining to the estimation of spatiotemporal and kinematic measures was presented, and a general overview of previous methodologies used for each stage of data processing was provided. For the estimation of spatiotemporal measures, which includes stride length, stride rate, and stance/swing duration, measurement thresholding and zero-velocity update approaches were discussed as the most common methodologies used to estimate such measures. The methodologies used for the estimation of joint kinematics were found to be broad, with the combination of Kalman filtering or complimentary filtering and various sensor to segment alignment techniques including anatomical alignment, static calibration, and functional calibration methods identified as being most common. The effect of soft tissue artefacts, device placement, biomechanical modelling methods, and ferromagnetic interference within the environment, on the accuracy and validity of IMC, was also discussed. Where a range of methods have previously been used to estimate human spatiotemporal and kinematic measures, further development is required to reduce estimation errors, improve the validity of spatiotemporal and kinematic estimations, and standardize data processing practices. It is anticipated that this technical summary will reduce the time researchers and developers require to establish the fundamental methodological components of IMC prior to commencing further development of IMC methodologies, thus increasing the rate of development and utilisation of IMC.

## 1. Introduction

Motion capture systems have been used extensively in biomechanics research to capture spatiotemporal measures of stride length, stride rate, contact time, and swing time and angular kinematic measures of joint angles. Such measures are commonly used in disease/condition diagnosis, injury prevention, and sport performance analysis [1–7]. The most common technologies used to collect human spatiotemporal and kinematic measures are three-dimensional (3D) optical, two-dimensional (2D) video, and electromagnetic based systems [8]. When motion capture data is collected in conjunction with data from force platforms, angular kinetics may also be modelled.

Three-dimensional optical motion capture (OMC) systems are often considered to be the gold standard method of motion capture; however, these systems are expensive and typically confined to a small capture volume within a laboratory environment [9, 10]. For a full body motion analysis, researchers are required to place up to 50 markers at anatomically specific locations, and a line of sight to each marker must be maintained by at least two cameras for each data frame throughout the movement [9]. Maintaining a line of sight to each marker throughout the movement is a major challenge when using 3D OMC as markers often become displaced and/or occluded when implements (such as boxes for manual handling assessments and bats, balls, or barbells for sporting assessments) are included in the movement analysis [9]. The displacement and/or occlusion of markers results in loss of data, increased measurement error, increased tracking time, and sometimes the inability to analyse a captured movement.

Two-dimensional (2D) video motion capture is a more affordable alternative to 3D OMC, requiring one or more video cameras with sufficient frame rate and video processing software such as the freely available software Kinovea (http://Kinovea.org, France) or Tracker (Open Source Physics). A number of drawbacks exist for 2D video motion capture. Multiple video cameras may be required for a full motional analysis. For example, for a running gait motion analysis, cameras may be required with views of the frontal and sagittal plane to capture joint varus/vulgus rotation and joint flexion/extension, stride length, stance duration, and swing duration, respectively. The high frame rate required to ensure accuracy when capturing fast movements (particularly sporting movements) result in large file sizes and extensive processing time. Both marker-based and marker-less 2D video motion capture rely on a line of sight of the participant throughout the movement and as such see similar occlusion limitations to 3D OMC [9]. Parallax error caused by the participant performing the movement at a nonperpendicular angle (out of plane) to the camera and perspective error caused by the participant moving toward or away from the camera are additional sources of error when using 2D video motion capture [11, 12].

Electromagnetic motion capture requires the participant to wear a specially designed suit of electromagnetic receiver sensors which receive electromagnetic waves from a base station transmitter located within the vicinity of where the movement is to be performed [8]. The receiver/transmitter network allows the position and orientation of the body to which the receiver sensors are attached to be determined within space [8]. Electromagnetic motion capture systems do not rely on line of sight measurements and thus do not encounter the problems of marker displacement and/or occlusion when implements are included in the motion analysis [8]. Low sampling rates currently make electromagnetic motion capture systems unsuitable for fast movements [8]. Motion capture often takes place at laboratory, clinical, or sporting facilities where equipment in the environment emit electromagnetic disturbance. Electromagnetic motion capture systems are susceptible to electromagnetic interference from the surrounding environment, causing potentially large errors in orientation estimations [8].

While each of these traditional motion capture methodologies have their own advantages and disadvantages, no single method is appropriate for all applications. Recent developments in inertial measurement unit (IMU) and magnetic, angular rate, and gravity (MARG) sensor technologies have resulted in researchers proposing the use of such devices to overcome many of the limitations of traditional motion capture systems, particularly when data needs to be collected outside of a laboratory.

Inertial devices have been used for human motion capture in the areas of athlete external load monitoring [13–15], activity classification [16–20], and spatiotemporal and kinematic analysis [4–6, 21]. The methodology of external load monitoring using inertial devices uses the raw output data of the IMU/MARG device (often accelerations) and thresholding techniques to determine the amount of exposure an athlete may have to various magnitudes of acceleration (external load) over the course of a training session, game/competition, or other relevant period of time such as a week, month, or year [15]. Such data is typically used to provide some insight into athlete performance, training adaptation, fatigue, and risk of injury [15]. Activity classification is used to identify movement patterns such as walking, running, stair ascent/descent, and lying in various positions over an extended period of time (hours or days). Machine learning techniques such as K-nearest neighbour, decision trees, support vector machine, logistic regression, and discriminant analysis are often used to classify these common activities of everyday living [17, 22]. Activity classification can provide clinicians with valuable information about the decline in health or independence of elderly living at home, the activity levels of persons living with conditions or diseases, or the detection of falls or accidents [20].

Inertial-based human spatiotemporal and kinematic analysis requires complex sensor fusion and pose estimation methodologies to process raw MARG data. Numerous studies have demonstrated good agreement when comparing spatiotemporal and kinematic measures derived from IMU and MARG based motion capture systems with gold standard 3D OMC systems in clinical, ergonomic, and sporting applications [4, 23–27]. Similar to traditional motion capture methods, researchers have suggested the accuracy of IMU and MARG based motion capture to be dependent on the algorithms and methodologies used to process the raw data captured by the device [28, 29].

Previous research and reviews have primarily focussed on either the overall validity of inertial-based motion capture (IMC) (excluding methodology considerations) [4, 8, 30, 31], sensor fusion methodologies [32, 33], or position and orientation estimation (pose) methodologies [34–38], making it difficult and time consuming for researchers and developers to piece together all essential methodological components. Two reviews have attempted to summarise the methodological components of IMC; however, these reviews have limited detail around critical considerations such as sensor fusion, pose estimation, soft tissue artifacts (STA), sensor placement, biomechanical modelling, and magnetic calibration, which should be made when developing an IMC solution [39, 40]. The following technical summary is aimed at providing background and reference on all methodological components which must be considered when implementing an IMC solution for a given application (Figure 1). Such a summary will reduce the time spent by researchers and developers establishing the fundamental methodological components of IMC prior to further developing current techniques and enhancing the rate of development and utilisation of IMC.

## 2. Sensor Fusion

The process of sensor fusion reduces the error inherent in the orientation estimation obtained from raw MARG data. The output of the sensor fusion step is used in subsequent steps of data processing toward the estimation of kinematic and spatiotemporal measures using IMC.

Inertial measurement units consist of an accelerometer and gyroscope to measure linear acceleration and angular rate, respectively. In addition to accelerometers and gyroscopes, MARG sensors include a magnetometer to measure magnetic field strength [41].

Integration of the angular velocity measured by the gyroscope provides an orientation estimation of the sensor at each time point relative to its initial orientation in the local frame. Integration of the gyroscope bias, which is inherent in the sensor at manufacture, leads to a slowly drifting (low frequency) cumulative error in the orientation estimation [33]. As the orientation is estimated in the local sensor frame, additional processing is required to establish a global reference frame, where a relationship between the orientation of each device in the network can be established [33]. This simplistic approach of integrating angular rate measures for device, and body orientation is insufficient for reliable human motion capture.

Accelerometers measure acceleration caused by gravity as well as acceleration caused by the motion of a body to which the sensor is attached. The measurement of acceleration due to gravity enables an estimation of the “up” direction (pitch and roll) of the sensor in the global reference frame [33]. The pitch and roll orientation estimation of the accelerometer may therefore be used to correct the pitch and roll component of the drift caused by the integration of the angular rate signal. Acceleration measurements are however corrupted by high frequency noise caused by movement of the sensor, leading to error in the pitch and roll orientation estimation when the sensor is in a non-quasi-static state [33].

Magnetometers measure the magnetic field strength of the Earth, enabling the definition of the Earth's horizontal North/East plane (heading or yaw) [33]. Similar to both the gyroscope and accelerometer, the magnetometer has its own inherent error in the orientation estimation. Ferromagnetic disturbances in the surrounding environment, causing the signal to be corrupt by high frequency noise, result in error in the orientation estimation by the magnetometer [41, 42].

Sensor fusion algorithms can be used to take advantage of the orientation estimation obtained by the gyroscope and the global references obtained by the accelerometer (pitch and roll) and magnetometer (yaw), while reducing the errors caused by the high and low frequency noise associated with each of the measures. The two most common methods of sensor fusion are the complementary filter [41, 43, 44] and the Kalman filter [45–47].

### 2.1. Sensor Fusion: Complementary Filter

A complementary filter is used to combine two measurements of a given signal, one consisting of a high frequency disturbance noise and the other consisting of a low frequency disturbance noise, producing a single signal output measurement [33]. Using filter coefficients/gains, the reliance on each input and response time for drift error correction can be manipulated, with shorter response times coming at the expense of greater output noise [33].

When applied to MARG data for orientation estimation, one such approach is to use a two-stage complementary filter to obtain a combined orientation estimation with a smaller error component than what could be obtained by using just a single sensor signal [48]. The application of a two-stage complementary filter can be briefly described as follows (see also Figure 2), with detailed derivation of complementary filter equations presented in Valenti et al. [48]:

- Orientation is estimated using accelerometer data
- Accelerometer orientation estimation is corrected based on a defined threshold adhering to the deviation from a known quantity (e.g., gravity). Correction is achieved using a gain to characterize the cut-off frequency of an applied filter
- The corrected accelerometer-based orientation estimation is fused with the low-frequency corrupt gyroscope-based orientation estimation, producing a complementary estimation of the device pitch and roll
- Magnetometer measures are examined for environmental ferromagnetic disturbances, and orientation estimation from the magnetometer data is corrected using a similar approach to the accelerometer-based orientation correction
- The pitch and roll (gravitational) orientation estimation is fused with the magnetometer yaw orientation estimation to provide a full attitude and heading orientation estimation

Although the accuracy of the orientation estimation and computational expense of the process can differ slightly between various complementary filter methodologies [41, 44], the complementary filter is generally computationally less expensive than other sensor fusion approaches [46, 49]. The low computational cost of the complementary filter enables the use of low power, wearable MARG devices, where data processing can be undertaken onboard the MARG device and streamed live for visualisation on external devices [41]. The smaller size of such wearable MARG devices may be particularly important for human motion capture where minimal disturbance to a person's natural movement is desired, enhancing the ecological validity of the analysis. The computational efficiency of the complementary filter however generally comes at the cost of the ability to tune the filter for a given application or environment, often resulting in an overall greater error in orientation estimation with reference to ground truth, when compared to sensor fusion approaches such as the Kalman filter [32, 46].

### 2.2. Sensor Fusion: Kalman Filter

The Kalman filter works on a prediction and correction process to estimate the state of a dynamic system from noisy measurements [49]. Various forms of the Kalman filter have been used for orientation estimation, with varying levels of complexity and assumptions being used in each solution [46, 51–53].

In its most simplistic form and using MARG data, five steps are typically employed in a Kalman filter-based solution for each time interval [52]:

- The a priori state estimate is obtained from the accelerometer, gyroscope, and magnetometer output measures
- The a priori error covariance matrix is established in an attempt to compensate for sensor bias and Gaussian measurement noise
- As the measurement model of the accelerometer and magnetometer is inherently nonlinear, a first order Taylor Maclaurin expansion of the current state estimate is performed by computing the Jacobian matrix
- Using the a priori state estimate, the a priori error covariance matrix and a set of measurement validation tests, an expression for the Kalman gain is established. The Kalman gain is used to give relative weight to either the current state estimate or the measurement
- An updated estimate (a posteriori) of the state estimate and error covariance matrix can then be computed

While these steps are generalisable to most Kalman filters, Figure 3 depicts, specifically, a block diagram of an indirect Kalman filter applied to MARG data [54, 55]. For brevity, state models and Kalman equations have been excluded from this paper; as such, the reader is directed to MEMS Industry Group [54] and The MathWorks Inc. [55] for further derivation of the particular case presented.

Although the Kalman filter is recognised for its greater tunability for a given application or environment and thus reduced error in orientation estimation when compared to the complimentary filter approach [32], the Kalman filter process is complex and requires high grade IMU and/or MARG sensors. The combination of high sampling rates (up to 30 kHz) required for the linear regression iterations, large state vectors, and additional linearisation through an extended Kalman filter make the Kalman filter based solution computationally expensive [41]. Where onboard processing is required for live visualisation of human motion, the physical size of the equipment required to satisfy these high computational demands may currently inhibit natural movement of the person wearing the device [41].

## 3. Pose Estimation

Orientation estimations of each IMU/MARG device obtained by means of sensor fusion must be further processed to obtain spatiotemporal and angular kinematic estimations of the human body. To estimate spatiotemporal and angular kinematic measures of the body, the position and orientation (pose) of the body/body segment must be established. Where both raw MARG data and sensor orientation estimation data (obtained as a result of sensor fusion) are typically used in this process, some of the processing methodologies used for angular kinematic estimations may also be required when establishing spatiotemporal estimations (namely, sensor to segment alignment).

### 3.1. Angular Kinematics

The placement of an IMU or MARG device on the segment immediately proximal and distal to a joint and taking the relative orientation of the two segments has been commonly proposed as a possible method of estimating joint angular kinematics [56]. The challenges associated with the estimation of joint angular kinematics using this method arise from the complexity of accurately estimating the device orientation using sensor fusion methods (as described previously) and the alignment of the sensor coordinate system to the corresponding segment coordinate system [57]. This process is commonly referred to as sensor to segment alignment. The three primary methods of sensor to segment alignment used in previous literature are the anatomical alignment, functional calibration, and static calibration methods. Most recently, deep learning techniques have also been used for sensor to segment alignment.

#### 3.1.1. Anatomical Alignment

The anatomical alignment method sees the alignment of the local rotational axes within the IMU/MARG device, with the anatomical axis of the body segment to which the device is attached [23, 24, 58, 59]. The relative rotation as estimated by the proximal and distal sensor for the aligned axes can then be assumed as the joint angle estimation throughout a movement. The advantage of the anatomical alignment method is seen in the use of the local (device) coordinate system for orientation estimation, thus not requiring any form of mathematical transformation from a local to a global coordinate system. The associated error and resultant overall accuracy of the joint angle estimation when using this method are highly dependent on the proper alignment of each device axes with the axes of the segment of interest [36, 59] and therefore may require the assistance of an experienced anthropometrist or specialised alignment equipment [60].

#### 3.1.2. Functional Calibration

Alignment of the local (device) coordinate frame with the segment coordinate frame has been achieved through functional calibration (FUNC) methods [61–63]. Functional calibration methods typically use predefined calibration movements and a set of assumptions (limiting the degree of freedom of a joint) to establish the average axis of rotation of a joint. Using the FUNC method, a MARG device may be arbitrarily placed on the limbs proximal and distal to a joint, and the orientation of each device in the global reference frame may be determined by an appropriate sensor fusion algorithm. With the two devices secured to the segments of a participant, the participant is asked to perform an isolated rotation about two single joint axes. For example, the first rotation may be about the longitudinal axis (i.e., internal/external rotation at the hip), while the second rotation may be about the medial/lateral axis (i.e., flexion/extension at the hip) [62]. Using numerical methods, the common axis of rotation can be determined, with the remaining axis of rotation assumed to be perpendicular to the two axes established from the movements [62].

The primary advantage of the FUNC method is in the ability to arbitrarily place sensors on each segment, thus eliminating the requirement of assistance of an experienced anthropometrist for sensor placement or additional alignment devices. Although the FUNC method has been further developed to be implemented with arbitrary movements [56], some clients may be unable to perform the required functional calibration movements [64]. Additionally, the numerical and optimization methods used to establish a common axis of rotation between segments are typically computationally expensive, resulting in the requirement of devices with greater processing capacity or off-board processing [56, 65, 66].

#### 3.1.3. Static Calibration

The static calibration (STAT) method is a somewhat hybrid approach of the anatomical alignment and FUNC methods. The STAT method requires a single axis of a “base” MARG device (typically located on the pelvis) to be aligned with a single axis (typically medial/lateral) of the segment [34, 67]. The advantage of this method is once one axis of a single sensor has been aligned with a segment axis; all MARG devices attached to other segments can be arbitrarily oriented.

A short, static, neutral calibration pose (five seconds) is captured to orient each sensor in the global frame using an appropriate sensor fusion algorithm. The vertical axis of the base MARG device is then corrected (rotated) to align with the gravity vector, leaving the remaining unknown (anterior/posterior) axis to be defined as being perpendicular to the medial/lateral and vertical axes [67]. This establishes an initial segment coordinate system in the global frame which may be used for all other segments, assuming all other segments were aligned during the calibration pose.

The arbitrarily aligned axes of the MARG devices attached to all other segments are then transformed to the initial segment coordinate system established from the base MARG using a mathematical transformation. Once the initial orientation of each segment in the global frame is known and thus can be tracked throughout a movement, a joint angle is calculated as the difference in orientation of two segments in the global frame.

As a somewhat hybrid approach, the STAT method provides the advantage of arbitrary device placement (except for the base unit) and relatively short computational times, when compared to FUNC methods. Similar to the anatomical alignment method, the STAT method assumes the accurate alignment of the single axis of the MARG device with a chosen axis of the base segment. As this is only a requirement for a single sensor/segment pair, the time taken by an experienced anthropometrist or trained person in assisting with the placement of sensors may be reduced. Where misalignment of the base sensor and/or misalignment of the participant body segments with a standard anatomical pose during static calibration is encountered, error in the sensor to segment alignment will occur.

#### 3.1.4. State-of-the-Art Deep Learning

To the author's knowledge, only one study has used state-of-the-art deep learning approaches for sensor to segment alignment in human motion capture [35]. The methodology used a set of both real and simulation data to train a model to identify the orientation of a MARG device attached to a body segment and to align the axes of the device with the anatomical axes of the corresponding segment. Sensors to segment alignment were performed for the pelvis and bilateral thigh, shank, and foot. Three datasets were used to train and test the model, with a final optimal model established using a combination of these datasets.

Dataset one consisted of real inertial data collected from 28 participants walking for six minutes in a figure eight pattern with a single inertial device orientation. Dataset two consisted of a sample of four participants walking back-and-forth in a 5 m line for one minute with nine different inertial device orientations. Dataset three consisted of simulation data established from a publicly available OMC dataset of 42 participants performing different walking styles. Inertial devices were mapped to the underlying model of dataset three using 64 alignment variations [35]. The final optimal model used datasets one, two, and three to train the model and a single participant from dataset two and a single participant from dataset three (not included in the training dataset) for testing. A mean alignment error of 15.21° was reported using the final optimal model, with a mean computational time for the training of such model of 48 hours [35].

Based on the results of Zimmermann et al. [35], deep learning methods appear to require a large set of training data and a large number of alignment variations to ensure reduced error and optimal sensor to segment alignment [35]. Although the development of the method of sensor to segment alignment using deep learning techniques is in its relative infancy, further development of the method may result in sensor to segment alignment using deep learning becoming common practice for IMC.

In addition to joint kinematic measures, researchers are often also interested in recording spatiotemporal measures for full gait analysis. Many of the data processing methods to achieve spatiotemporal measures using IMC build on and rely upon the assumption of sensor to segment alignment.

### 3.2. Spatiotemporal

While gait event detection such as heel strike and toe-off and subsequent spatiotemporal parameters such as swing and stance duration and cadence may be identified through various relatively simple threshold approaches using measures of angular rate and linear acceleration [68], estimation of stride length is typically more complex [69, 70]. Two approaches for stride length estimation have primarily been used in previous literature: the biomechanical modelling [71–73] and strap-down integration approach [74].

In the biomechanical modelling approach, the lower limbs are typically modelled by means of a double pendulum [71–73]. Such modelling approach is, however, restricted to the analysis of movement in the sagittal plane, limiting the accuracy of the method for stride length estimation of persons with irregular gait patterns [74, 75]. Although not free from its own challenges, the strap-down integration approach enables multiplanar analysis, and as such, will be the focal method for spatiotemporal estimation in this technical summary [74].

Assuming sensor to segment alignment has been implemented on a foot/shoe mounted MARG sensor, double integration of the raw acceleration measures, after the subtraction of acceleration due to gravity, theoretically provides an estimation of the distance travelled throughout a given movement duration. Integration of the high frequency noise within the acceleration measure results in a cubically growing positional error [74]. The strap-down integration approach, by means of zero-velocity update (ZUPT), has been generally accepted as the most robust approach to overcome the propagation of error caused by integration of acceleration data for position estimation [69]. The ZUPT algorithm has seen multiple variations [69, 70, 74, 76, 77] and typically relies on the accurate identification of the stance phase of the gait cycle (where the foot momentarily experiences zero velocity relative to the ground) so to “reset” the cubically growing error caused by the double integration of noisy raw linear acceleration data [69, 74, 78, 79].

Thresholding techniques have been used to identify phases of a gait cycle, whereby the resultant angular velocity of the foot is monitored for zero angular rotation about any axis throughout the stance phase [80]. Although the exact value of zero angular rate may not be reliably captured in real life, setting a threshold of, for example, 1 rad/s has been suggested to reliably capture the stance phase during walking [80]. For running or other higher velocity movements where the duration of the stance phase is shorter than walking, the threshold value will likely require adjustment, or the addition of other measurements to the logic statement may be required [70, 81]. The use of both foot angular velocity and orientation data has been demonstrated as a possible method of identifying instances of heel strike and toe-off during a gait cycle [68]. Using this method, toe-off may be identified by searching for the first maximum in angular velocity within a specified search window spanning peak ankle plantar flexion. Similarly, heel strike may be identified by searching for the zero angular velocity crossing point within a search window spanning peak ankle dorsiflexion [68]. Search window sizes should be set specific to a given movement (e.g., walking, running, and pathological gait pattern), with the most appropriate window sizes typically achieved through an iterative process.

As the sensor orientation is transformed from the sensor frame to the navigation or global frame, the acceleration due to gravity can be removed, leaving just the acceleration due to the motion of the sensor. The remaining motional acceleration can then be integrated to give the estimated velocity of the sensor. Where the stance phase (zero velocity) has previously been identified through the identification of heel strike and toe-off events, the integrated velocity and thus measurement error is “reset” to zero [80]. By resetting the velocity to zero during each stance phase, the drift error is limited to the relatively short duration of a stride. The corrected velocity may then be once again integrated to give position, where stride length is the difference in position between two consecutive stance phases.

The use of Kalman filtering techniques can improve the accuracy of the described naïve ZUPT approach [70]. Instead of resetting the velocity to zero where a stance phase is identified, the Kalman filter uses an error state vector consisting of biases for acceleration, angular rate, attitude, velocity, and position to reset velocity and position to an estimated near-zero value [70, 77].

Although the gait event detection and ZUPT methods described in this summary are a general overview of methods used in previous literature, an example of how a selection of these methods may fit together to estimate gait spatiotemporal parameters is provided in Figure 4. The reader is directed to Jasiewicz et al. [68] and Fischer et al. [70] for further implementation details.

## 4. Additional Considerations

Aside from selecting the most appropriate sensor fusion and pose estimation processing methodologies for a given application, other components of the methodological design such as device placement, biomechanical modelling methods, and magnetometer calibration also warrant consideration so to minimize the propagation of errors and optimize the accuracy of an implemented IMC methodology.

### 4.1. Device Placement

Soft tissue artefacts (STA) are suggested to be a significant source of error when measuring human kinematics using OMC methods [82]. Soft tissue artefacts occur when the skin (and underlying adipose tissue and muscle) to which the markers/sensors are attached, move relative to the bone for which the orientation and kinematics of the body is being estimated [82]. Inertial-based motion capture is also not exempt from the error caused by STA. Where OMC methodologies often use rigid clusters of markers [83] and/or anatomical modelling assumptions [84] to reduce the effects of STA, research into the reduction of STA effects on IMC is limited [85, 86]. Frick et al. presented a two-part study using numerical methods to reduce the effect of STA on inertial-based joint centre estimations. The method used a single frame optimization (SFO) algorithm to determine the location and orientation of the joint centre relative to the sensor at each time frame. Although the method showed good agreeance with state-of-the-art OMC joint centre estimations on a mechanical rig, the SFO cost function assumes the joint centre to be undergoing negligible acceleration, which may be violated for many applications. The method proposed by Frick and Rahmatalla [85] demonstrates the potential in the reduction of STA when using IMC methods; however, further development is required before the SFO method is considered a practical solution for more complex applications [85, 86].

Spatiotemporal parameters such as stride length, stride time, and contact time have regularly been obtained from a single IMU/MARG device worn on the pelvis, ankle, or foot [1, 2, 87, 88]. The validity of these IMU/MARG derived spatiotemporal measures has been suggested to be affected by the location of the device [89]. When compared to ankle and pelvis worn IMU/MARG devices, foot mounted IMU/MARG devices have been found to result in greater validity of spatiotemporal estimations [87, 88]. Positioning the device closer to the source of impact (ground) may result in less signal attenuation from STA and naturally occurring shock absorption by proximal segments and thus greater accuracy in gait cycle event detection (such as heel strike, midstance, and toe-off) [2, 90].

### 4.2. Biomechanical Modelling

Often considered a gold standard, OMC typically combines anatomical assumptions and anatomical marker locations to estimate joint angle kinematic measures using modelling techniques (modelled measures) such as the Plug-in Gait model (Oxford Metrics, Oxford, UK). Inertial-based motion capture typically relies on the unmodelled relative orientations of a proximal and distal sensor to a joint for joint angle estimation [6]. Due to these differences in modelling assumptions, the modelled measures obtained from OMC are expected to differ somewhat from the naïve relative joint angles commonly obtained using IMC [6, 91].

Brice et al. [6] compared IMC relative joint angles with OMC relative angles (unmodelled with reflective markers attached to the inertial device) and IMC relative joint angles with OMC modelled measures for the pelvis and torso in the sagittal, frontal, and transverse plane. Participants performed three sets of a self-selected slow and two sets of self-selected fast rotation of the torso relative to the pelvis in each anatomical reference plane. Good agreement was reported between the IMC relative joint angles and the OMC relative angles (RMSE%: 1–7%). Less agreement was reported between the IMC relative joint angles and OMC modelled measures (RMSE%: 4–57%). Similar results to Brice et al. [6] have been found by Cottam et al. [91] for pelvis, thorax, and shoulder joint angles during cricket bowling. No significant differences were reported between IMC and OMC relative angles; however, significant differences in shoulder rotation, thorax lateral flexion, and thorax to pelvis flexion-extension and lateral flexion were reported between IMC relative joint angles and OMC modelled joint angles at various stages of the cricket bowling delivery stride [91].

The results of Brice et al. [6] and Cottam et al. [91] suggest that IMC is capable of accurately measuring pelvis and torso relative angles during slow and fast multiplanar movements; however, these relative angles may not be representative of or directly comparable to those of an OMC system where anatomical modelling is used to estimate joint angles. It has recently been suggested that the joint kinematics measured using both OMC and IMC methods may not represent the true kinematics of the joint due to the underlying assumptions made when using each method [25, 27, 30]. Further development of OMC and IMC modelling techniques may be required to enable valid comparison between OMC and IMC joint angle estimations, with development of each method being further extended to achieve a greater representation of the true kinematics of the joint.

### 4.3. Magnetometer Calibration

Although the inclusion of a magnetometer in an IMC system allows the definition of the orientation of the MARG device in a global North, East Down (NED) reference frame, such global orientation estimation may be corrupted by ferromagnetic disturbances within the environment. Often, the validation of IMC systems occurs within a laboratory environment where gold standard systems (such as OMC systems) are situated and used for comparison. Measurement equipments within a laboratory, as well as structural iron in the flooring, walls, and ceiling of the building have proven to be a considerable source of ferromagnetic interference [92]. When using MARG devices for motion capture within such environments, a magnetic calibration of each MARG device is recommended [92].

Magnetic calibration procedures reduce the effect of hard iron effects (fixed bias with respect to the local reference frame of the sensor) and soft iron effects (variable distortion dependent on the orientation of the sensor) [42]. In an undisturbed environment, the magnetic field strength data of a magnetometer rotated through a full range of 3D rotation should form a perfect sphere centred around some origin. Ferromagnetic disturbances distort this ideal spherical formation of data to the extent of an ellipsoid shape (due to soft iron effects) and shift the centre of the ellipsoid away from the origin (due to hard iron effects). To correct for hard and soft iron effects, a best fit ellipsoid is established using parameter solving algorithms in an attempt to form a spherical representation of the raw data (Figure 5) [42].

Performing movements > 40 cm above ground level, starting data capture in an area of low ferromagnetic disturbance and ensuring sufficient capture time before commencing the movement to allow the sensor fusion Kalman filter to compensate for ferromagnetic disturbances have also been shown to reduce error in orientation estimation caused by ferromagnetic disturbances [92]. At minimum, researchers and developers should attempt to correct for yaw estimation error caused by hard iron effects, and where appropriate implement, the aforementioned additional strategies based on the environment in which the IMC system will be used.

### 4.4. Error Propagation

The error associated with each stage of data processing propagates toward a total IMC system error. For example, the combined error in a single body segment orientation estimation is the sum of the sensor fusion error, the sensor to segment alignment error, and any additional error caused by STA or biomechanical modelling assumptions. Where the goal may be to estimate the relative orientation between two segments (joint angle), the error in each body segment orientation estimation is once again combined. Careful implementation and further development of the data processing and error minimization strategies presented throughout this technical summary will contribute to the reduction in total system error and resultant overall accuracy of IMC systems.

## 5. Conclusions and Recommendations

Inertial-based motion capture addresses many of the limitations associated with traditional motion capture systems including marker occlusion and dropout, expensive equipment costs, and the ecological validity of performing movements in a confined laboratory environment. The accuracy of IMC systems is suggested to be primarily dependent on the data fusion algorithms and pose estimation methodologies used to interpret human motion from raw MARG data. Additionally, the effect of soft tissue artefacts, device placement, biomechanical modelling methods, and ferromagnetic interference within the environment should be carefully considered to enhance the accuracy and validity of MARG derived spatiotemporal and kinematic estimations.

## Figures and Tables

**Figure 1:** Workflow of IMC and where sections of this technical summary lay within the general methodological structure.

**Figure 2:** Complimentary filter approach example (adapted from Wu et al. [50] and Valenti et al. [48]).

**Figure 3:** Kalman filter approach example (adapted from MEMS Industry Group [54] and The MathWorks Inc. [55]).

**Figure 4:** Zero-velocity update approach example (adapted from Jasiewicz et al. [68] and Fischer et al. [70]).

**Figure 5:** Magnetic calibration approach example (adapted from Ozyagcilar [42]).

## Data Availability

No data were used to support this study.
